# Convolutional Neural Network in Microsurgery Treatment of Spontaneous Intracerebral Hemorrhage

**DOI:** 10.1155/2022/9701702

**Published:** 2022-08-09

**Authors:** Xiaoqiang Wu, Dan Chen

**Affiliations:** ^1^Department of Neurosurgery, The People's Hospital of Sixian, Sixian, Anhui Province 234399, China; ^2^Department of Neurosurgery, The Third People's Hospital of Hefei, Hefei 230022, China

## Abstract

**Objective:**

To explore the convolutional neural network (CNN) method in measuring hematoma volume-assisted microsurgery for spontaneous cerebral hemorrhage.

**Methods:**

A total of 120 patients with spontaneous cerebral hemorrhage were selected and randomly divided into control and CNN groups with 60 patients in each group. Patients in the control group received traditional Tada formula to calculate hematoma volume and microsurgery. Convolutional neural network algorithm segmentation was used to measure hematoma volume, and microsurgery was performed in the CNN group. This article assessed neurological function, ability to live daily, complication rate, and prognosis.

**Results:**

The incidence of postoperative complications in the CNN group (13.33%) was lower than the control group (43.33%). The neurological function and daily living ability in the CNN groups were recovered better. The incidence of poor prognosis in the CNN group (16.67%) was lower than the control group (30.00%).

**Conclusion:**

Convolutional neural network measurement of hematoma volume to assist microsurgical treatment of spontaneous intracerebral hemorrhage patients is conducive to early recovery, reducing the damage to the patients' cerebral nerves.

## 1. Introduction

Spontaneous intracerebral hemorrhage is one of the most common critical and severe diseases in neurosurgery, which occurs in middle-aged and elderly patients [1–3]. It is a cerebrovascular disease with high mortality and disability rate. For a long time, researchers have conducted a lot of research and practice on the pathogenesis and treatment of spontaneous intracerebral hemorrhage. In recent years, under the influence of various factors such as life pressure and diet, the incidence of spontaneous intracerebral hemorrhage shows a significant upward trend [4], and the onset age gradually decreases, seriously impacting patients and families, and society.

Spontaneous intracerebral hemorrhage is a hemorrhage in the brain parenchyma that extends into the ventricle or subarachnoid space [1]. Although the rapid development of modern medical science and technology and the continuous development of minimally invasive surgical techniques and equipment provide new methods for the treatment of hypertensive intracerebral hemorrhage, the total mortality of intracerebral hemorrhage is still very high. Hematoma volume was a determinant of mortality within 30 days [5].

Due to the high incidence, disability, and mortality of spontaneous intracerebral hemorrhage, timely and effective treatment of hypertensive intracerebral hemorrhage is required. Accurate measurement of intracerebral hemorrhage is essential for clinical treatment and evaluation of curative effects. CT is the first choice for cerebral hemorrhage. Tada formula is a traditional method for measuring intracerebral hemorrhage, which is simplified from the elliptic sphere volume formula [6]. Its premise is that the hematoma is approximately regular elliptic sphere. However, the clinical hematoma is often irregular in shape, resulting in low accuracy of Tada formula measurement results and poor repeatability due to the influence of subjective factors [7, 8].

With the development of deep learning and other computer technologies [9–11], more and more scholars are using relevant technologies to calculate hematoma volume [12–14]. Yu et al. [15] constructed a deep learning algorithm covering hematoma volume of all types of intracerebral hemorrhage, which has higher accuracy and consistency with manual segmentation method. This study analyzed the segmentation method based on the convolutional neural network (CNN) algorithm to calculate hematoma volume and microsurgery to treat spontaneous intracerebral hemorrhage.

## 2. Materials and Methods

### 2.1. General Information

The study lasted from May 2018 to April 2021. A total of 120 patients with spontaneous intracerebral hemorrhage were selected and randomly divided into control group and CNN group (60 cases equally) according to a random number table method. The male-female ratio and the hemorrhage location in the control group and CNN group are shown in Figure 1. The two groups found no significant difference between gender, age, bleeding site, and other general information (*P* > 0.05, Table 1).

### 2.2. Selection Criteria

Inclusion criteria were as follows: (1) signed the informed consent for the study approved by the hospital ethics committee, (2) met the diagnostic criteria for cerebral hemorrhage and had a clear history of hypertension, (3) the first onset of hypertensive intracerebral hemorrhage, (4) intracranial hemorrhage was confirmed by craniocerebral CT examination, and (5) the amount of blood loss was 30~70 mL.

Exclusion criteria were as follows: (1) intracerebral hemorrhage caused by autoimmune diseases or coagulation disorders, (2) cerebral hemorrhage caused by vascular diseases such as aneurysm, (3) cerebral hemorrhage caused by brain trauma, inflammation, and dilated pupil requiring decompression by bone flap removal and anticoagulant drug treatment, and (4) patients with incomplete case data or unable to achieve a long-term follow-up.

### 2.3. Experimental Grouping

The overall structure of this experimental process is shown in Figure 2.

#### 2.3.1. Control Group

Preoperative hematoma volume was calculated by 2 doctors with 3 years of neuroimaging diagnosis experience according to Tada's formula, which is as follows:

(1) $$\begin{array}{c} V\left(\text{bleeding}\right)=\frac{A\times B\times C}{2}. \end{array}$$

The ABC/2 volume formula can express the Tada volume formula. The bleeding area of each section was compared with the maximum section. The amount of bleeding and the physician's measurement time were recorded.

A craniotomy was performed. Before the operation, the hematoma was located according to the results of cranial CT imaging, craniotomy was routinely performed, and the hematoma was removed under the microscope. Postoperative imaging review was performed.

#### 2.3.2. CNN Group

In order to reduce the overfitting risk of constructing algorithm segmentation results, we have included a large number of cerebral hemorrhage cases in the early stage and evaluated the performance of the algorithm model through the interactive brain image segmentation algorithm (Figure 3).

When the CNN algorithm analyzes the image, the image is deaveraged, as shown in the following equation:

(2) $$\begin{array}{c} a^{*}=a-\lambda , \end{array}$$

where *λ* is the average of the image set and *α* is the eigenvalue.

The complete CNN includes many layers. The convolutional layer is the most crucial part and can be described by the following equation:

(3) $$\begin{array}{c} a_{j}^{l}==e\left(\underset{i}{\sum }\in N_{j}a_{j}^{l-1}\times h_{ij}^{l}+d_{j}^{l}\right). \end{array}$$

The pooling layer can be described as follows:

(4) $$\begin{array}{c} a_{j}^{l}=\text{down}\left(a_{j}^{l?1}\right). \end{array}$$

Since the CNN algorithm has a good feature extraction performance, we performed fusion preprocessing on CT images and automatically detected and segmented hematoma area on the images by CNN algorithm (Figure 4).

According to the measurement results, craniotomy was performed, and the removal of craniotomy hematoma was performed under the microscope. Imaging review was performed after surgery.

### 2.4. Evaluation Index

#### 2.4.1. Complications

In this paper, the incidence of postoperative complications was observed and counted as in the following equation:

(5) $$\begin{array}{c} C=\frac{I+R+CR+SC}{T}\times 100\%. \end{array}$$

In Equation (5), *C* represents complications. It is formed by the sum of *I* (infection), *R* (rebleeding), *CR* (cerebral infarction), and *SC* (stress ulcer).

#### 2.4.2. Nerve Function

Neurological function was assessed by the National Institutes of Health Stroke Scale (NIHSS) before and 3 and 6 months after surgery.

#### 2.4.3. Daily Living Ability

The ability of daily living (ADL) was used to evaluate the daily living ability of 2 groups in the same time point.

#### 2.4.4. Poor Prognosis

The outcomes were followed up for 6 months by the Glasgow Outcome Scale (GOS). The adverse outcomes (*P*) are formed by the sum of *I* (disease death, 1 point), *PS* (plant survival, 2 points), and *SM* (severe disability, 3 points).

(6) $$\begin{array}{c} P=\frac{I+PS+SM}{T}. \end{array}$$

### 2.5. Statistical Methods

SPSS 23.0 statistical software was used for data processing and analysis. The comparison of between groups was performed by independent sample *T*-test. A group design and a two-sample comparison were used to compare the hierarchical grouped data.

## 3. Results

### 3.1. Complications

The total proportion of postoperative complications in the CNN group (13.33%) was significantly lower than that in the control group (43.33%) (Table 2).

### 3.2. Neurological Function and Daily Living Ability

There was no significant difference in preoperative neurological function and daily living ability between the two groups, but 3 and 6 months after surgery, the neurological function and daily living ability of the two groups were better than those of the three groups before surgery (Table 3).

### 3.3. Poor Prognosis

The incidence of poor prognosis in the CNN group (16.67%) was lower than that in the control group (30.0%, Figure 5).

## 4. Discussion

The basic cause of disability and death caused by spontaneous intracerebral hemorrhage is the injury of brain tissue caused by acute intracerebral hemorrhage, intracerebral mass effect, cerebral edema, and cerebrospinal fluid circulation system obstruction, resulting in acute intracerebral pressure increase [16]. Therefore, in the clinical treatment of spontaneous cerebral hemorrhage, the timely and accurate evaluation of the bleeding volume and the effective removal of the intracerebral hematoma is the key to the treatment. Timely intervention can reduce the surrounding brain tissue after brain hematoma removal by oppression, ease the cerebrospinal fluid circulation obstruction, reduce secondary brain edema, reduce mortality, and improve survival quality.

The amount of bleeding in patients with spontaneous intracerebral hemorrhage is closely related to clinical treatment strategy, brain function recovery, and mortality [17]. The untimely and inaccurate measurement will affect clinical decision-making, delay the optimal treatment timing, and affect the therapeutic effect [18]. Therefore, accurate measurement of intracerebral hemorrhage has essential clinical significance [19]. CT quantitative method, Tada formula method, and stereology method are recommended to calculate the amount of cerebral hemorrhage in the 2006 guidelines for the surgical treatment of craniocerebral trauma in the United States. The CT quantitative method, also known as computer-assisted volume analysis (CAVA), is the gold standard for noninvasive measurement of intracranial hematoma volume, which has the advantages of accurate measurement and is not limited by bleeding shape [20, 21]. Equipment conditions limit the disadvantage, need to be completed on the CT machine, are time-consuming, and are not suitable for clinical emergencies. Tada formula is more accurate in measuring morphologically regular intracerebral hemorrhage. However, there are large errors for irregular intracerebral hemorrhage and manual segmentation is time-consuming and laborious [22, 23]. Stereology has made progress in measuring irregular hematoma, but it requires tools and is complicated.

This is a challenge for clinicians in order to grasp the condition better and more accurately answer clinical questions, especially in cases where traditional calculations of hematoma volume are inaccurate. Artificial intelligence technology's in-depth application in clinical medicine allows intracranial hematoma to be accurately and conveniently separated [24, 25]. This study explored the feasibility of using a convolutional neural network to calculate hematoma volume as a surgical indication.

The comparison of experimental data showed that the CNN group was superior to the control group in all indicators, with statistically significant differences among the groups (*P* < 0.05). Compared with the control group, the complications in the CNN group were lower. The neurological function and daily living ability were better before and after operation, and the incidence of poor prognosis was low.

Our results show that convolutional neural network calculation of hematoma volume guiding craniotomy treatment can reduce the incidence of postoperative complications and poor prognosis, reduce neurological impairment, but also help improve patients' daily living ability. We believe that convolutional neural network-based hematoma volume calculation has the advantages of timeliness, accuracy, and ease of operation [26]. Thus, the patients can obtain timely and effective treatment in a short time.

## 5. Conclusions

In conclusion, in the surgical treatment of patients with spontaneous intracerebral hemorrhage, the application of convolutional neural network to calculate hematoma volume as the reference of surgical indication has obvious advantages, which can significantly improve the prognosis of patients. At the same time, it is helpful to reduce surgical trauma, reduce complications, and promote the recovery of patients' neurological function.

## Figures and Tables

**Figure 1:** Male-female ratio and hemorrhage location in the control and CNN groups.

**Figure 2:** The overall structure of experimental process.

**Figure 3:** Schematic diagram of interactive brain image segmentation algorithm.

**Figure 4:** The CT images were preprocessed by the CNN algorithm.

**Figure 5:** Comparison of outcomes after 6 months of follow-up.

**Table 1:** Age and hematoma volume in the control and CNN groups.

Group	Age range (years)	Average age (years)	Hematoma volume (mL)
Control group	39-80	60.8 ± 1.9	40.2 ± 10.8
CNN group	41-82	61.2 ± 2.1	39.3 ± 11.1

**Table 2:** Comparison of complications between the two groups.

Group	Postoperative infection	Bleeding again	Stress ulcer	Cerebral infarction	Total incidence
Control group	5	6	5	10	26 (43.33)
CNN group	1	2	2	3	8 (13.33)
*χ* ^2^					22.16
*P*					<0.01

**Table 3:** Comparison of nerve function and ability of daily living.

Group	Nerve function			Ability of daily living		
	Preoperative	3 months after surgery	6 months after surgery	Preoperative	3 months after surgery	6 months after surgery
Control group	23.59	19.07	14.36	51.23	70.74	79.67
CNN group	24.11	10.47	8.66	50.38	81.08	91.32

## Data Availability

The data used to support the findings of this study are available from the corresponding author upon request.
